This article has been retracted.

# Protective Properties of the Extract of Chrysanthemum on Patients with Ischemic Stroke

**DOI:** 10.1155/2021/3637456

**Published:** 2021-11-30

**Authors:** Zhuoying Zhu, Shuxia Qian, Xudong Lu, Congying Xu, Yanping Wang, Xiaoling Zhang, Xin Yu, Yufei Shen

**Affiliations:** ^1^Institute of Neurology, The Second Affiliated Hospital of Jiaxing University, Jiaxing 314000, China; ^2^Bengbu Medical College, Bengbu 233000, China

## Abstract

Investigation of the protective effect of chrysanthemum extract in ischemic strokes patients is among the challenging issues with the traditional hospital system in general and smart technology-based hospitals in particular. In this study, we have evaluated the protective effect of chrysanthemum extract on patients with ischemic stroke by detecting the severity of stroke, neuronal indexes, and oxidative stress biomarkers. For this purpose, forty-six patients with ischemic stroke were randomly divided into the control group (*n* = 30) and chrysanthemum group (*n* = 30). The control group received standard stroke treatment, and the chrysanthemum group was treated with chrysanthemum extract 400 mg/day (200 mg/day, twice/day) on the basis of standard treatment. The groups were compared the effect of saffron capsules using the National Institute of Health Stoke Scale (NIHSS), serum neuron specific enolase (NSE), S100, brain-derived neurotrophic factor (BDNF), malondialdehyde (MDA), Su-peroxide dismutase (SOD), and total antioxidant capacity (TAC ) levels, at the time of first day and fourth day after treatment. On the first day after treatment, there was no significant difference in the NIHSS score, serum NSE, S100, BDNF, MDA, SOD, and TAC levels between the chrysanthemum group and the control group (*P* > 0.05). On the fourth day after treatment, the NIHSS, serum NSE, S100, and MDA levels were significantly reduced in the chrysanthemum group compared to the control group, while the BDNF, SOD, and TAC levels were higher (*P* < 0.05). In addition, compared to the levels on the first day, the NIHSS, serum NSE, S100, and MDA levels were significantly reduced, and the BDNF, SOD, and TAC levels were increased in the chrysanthemum group on the fourth day (*P* < 0.05). Chrysanthemum extract has the effects of scavenging oxygen free radicals and antioxidation and has a neuroprotective effect on ischemic stroke patients.

## 1. Introduction

Stroke, commonly known as cerebrovascular accident, is a series of cerebrovascular diseases which is caused by cerebrovascular rupture or cerebrovascular blockage [1, 2]. The traditional definition of stroke is based on clinical manifestations, and the clinical characteristic is the sudden loss of neurological function due to infarction or bleeding in the corresponding brain region [3, 4]. Stroke is one of the most common cerebrovascular diseases, with high mortality and disability rate, which has seriously threatened human health [5]. Among all stroke patients, ischemic stroke patients account for more than 80% [6]. The clinical symptoms are sudden fainting, numbness of lateral limbs, deviation of mouth angle and aphasia, and hemiplegia or even life-threatening in severe cases [7–9]. In the process of cerebral ischemia, it will stimulate oxidative stress response, a series of inflammatory reactions and release neurotoxins, resulting in serious damage to patients' neurons [10–12]. Therefore, improving oxidative stress and neuroprotection play an important role in the treatment of ischemic stroke.

Herbal medicines derived from plant extracts with natural antioxidant and pharmacological activities are being increasingly utilized to treat a wide variety of clinical diseases. Chrysanthemum is a species of perennial plant from the Asteraceae family and one of the most important ornamental flowers in the world [13]. Chrysanthemum is able to improve eyesight and prevent fatigue [14]. Chrysanthemum may be used to treat wind-heat type common cold, headache and dizziness, red and painful eyes, and toxin-induced swelling [15, 16]. The main ingredients of *Chrysanthemum morifolium* are volatile oils, flavonoids, chlorogenic acid, polysaccharides, phenols, and trace elements [17–19]. Flavonoid compounds, triterpenoids, and volatile oils are the main active components [20].

It has been reported that flavonoids from *Chrysanthemum morifolium* may significantly improve the activity of antioxidases in the tissues of rats with lead poisoning, relieve lipid peroxidation, and antagonize oxidative injury of the brain, liver, and kidney [21]. However, the mechanism of chrysanthemum extract in ischemic stroke is not clear. Therefore, further clinical studies are needed to clarify its role in ischemic stroke. In present study, we evaluated the protective effect of chrysanthemum extract on patients with ischemic stroke by detecting the severity of stroke, neuronal indexes, and oxidative stress biomarkers.

In this study, we have evaluated the protective effect of chrysanthemum extract on patients with ischemic stroke by the treatment of ischemic stroke.

For this purpose, forty-six patients with ischemic stroke were randomly divided into the control group (*n* = 30) and chrysanthemum group (*n* = 30). Likewise, a simplified classification approach is presented to divide patients into either selected or not selected groups.

The main contributions of this manuscript to the scientific community are given as follows.

- To evaluate the protective effect of chrysanthemum extract in ischemic strokes patients to improve the treatment process of this disease
- A sophisticated classification-based mechanism is developed to detect and predict, preferably at the earliest possible stage, severity of stroke, neuronal indexes, and oxidative stress biomarkers
- A technology-assisted classification approach is proposed, which has the capacity to separate suitable or appropriate patients from others

The remaining study is organized as follows. The proposed model and experimental device are shown in Figure 1. In subsequent section, a detailed description and analysis of the proposed method is presented, which is followed by a comprehensive analysis of the proposed method and its effectiveness in resolving the aforementioned issues. Experimental results are thoroughly examined and explained with proper justification in the experimental results section. Finally, concluding remarks and future direction are given.

## 2. Proposed Methods

In this section, a detailed and comprehensive description along with possible analysis is presented. Moreover, how patients are selected and not selected, which criteria is used? These questions are answered in this section.

### 2.1. Patients

Forty-six patients with ischemic stroke participated in this study, who had been referred to the Second Affiliated Hospital of Jiaxing University specifically between August 2018 and December 2020. All patients were diagnosed as ischemic stroke by brain computed tomography (CT) scan or magnetic resonance imaging (MRI). All patients were randomly divided into the control group and chrysanthemum group, with 23 cases in each group. Both groups received the standard treatment recommended by the guidelines of ischemic stroke during the study [18]. Standard treatment includes statins, aspirin, warfarin, ticlopidine, clopidogrel, and dipyridamole. The control group only received standard treatment, and the chrysanthemum group received chrysanthemum extract at the dose of 400 mg/day (200 mg/day, twice/day) on the basis of standard treatment. The chrysanthemum extract was purchased from Shaanxi Jinhe Biotechnology Co., Ltd. The present study was approved by the ethics committee of our hospital. All patients were hospitalized for more than fourth days. All patients and their relatives completed and signed an informed consent form.

### 2.2. Inclusion and Exclusion Criteria

Inclusion criteria [19]: the patients' NIHSS scores between 5 and 20 on admission and less than 24 h since the onset of the stroke. Patients and their relatives agreed to participate in the present study.

Exclusion criteria [20]: patients with medication intolerance, hemorrhagic stroke, NIHSS >20 during hospital stay, acute or chronic kidney failure (stages 4 and 5), acute liver failure or active liver disease (failure stages B and C), history of disability prior to the current stroke, acute ischemic heart stroke in the last 48 h, history of Alzheimer's disease or other types of dementia, the use of medications with possible neuroprotective properties in the last six months, receiving thrombolysis medication (tPA), central nervous system (CNS) tumor, and recent head trauma were excluded.

### 2.3. Blood Sample Collection

We collected blood samples from all patients on the first and fourth day after treatment. After clot forming, the serum was separated from the coagulated blood by centrifugation at 1000 g for 10 min at 4°C. Samples were then transferred into 0.5 mL microtubes and stored at −80°C.

### 2.4. NIHSS Scores

NIHSS scores [21] were performed on the day of admission and on the first day and the fourth day of treatment. Scores are calculated based on the examination of various neurological items and categorized as mild (1–4), moderate (5–15), moderate to severe (16–20), and severe (21–24). Two doctors scored independently.

### 2.5. Serum Levels of S100, NSE, BDNF, MDA, SOD, and TAC

In the present study, blood samples were taken on the first and fourth day after treatment, and patients' serum NSE, S100, BDNF, MDA, SOD and TAC levels were assessed. In order to measure serum NSE, S100, BDNF, MDA, SOD, and TAC levels, blood samples were centrifuged and immediately stored at −20°C to prevent the degradation of proteins. NSE, S100, and BDNF levels were evaluated in serum samples by using enzyme-linked immunosorbent assay (ELISA) kit (DRG NSE kit, Cat. Nr EIA 4610), (ZellBio GmbH, Cat No: ZB-13074S-H9648) and (ZellBio GmbH, Cat. No: ZB-1302-H9648). MDA level as an indicator of lipid peroxidation was determined by condensation with thiobarbituric acid at 532 nm using Teb Pazhouhan Razi Company kit (Tehran, Iran). SOD activity was measured based on the inhibition of the reduction of nitroblue tetrazolium by superoxide at 560 nm. TAC was measured by the ferric reducing/antioxidant power (FRAP) method using commercially available kit (ZellBio GmbH, Germany).

### 2.6. Statistical Analysis

SPSS 19.0 software was used for data statistical analysis (SPSS Inc., Chicago, USA) in the present study. The counting data were expressed in the form of *n* (%), and the data were analyzed by the chi-square test. The measurement data are tested by Kolmogorov–Smirnov to see whether the data conform to the normal distribution. The data conforming to the normal distribution are expressed in the form of mean ± SD, and the data are analyzed by the *t*-test. The data that do not conform to the positive distribution are expressed in the form of *M* (Q25, Q75) and use the Mann–Whitney *U* test. The two-way ANOVA analysis was used to compare the indexes on the first and fourth day of treatment, and *P* values less than 0.05 were considered significant.

## 3. Experimental Results and Observations

In this section, numerous experimental results obtained are compared with state-of-the-art existing methods, and the effectiveness of the proposed approach is resolving the challenging issue, i.e., detection of chrysanthemum extract in ischemic strokes patients specifically in the traditional hospital system.

### 3.1. Clinical Characteristics of Stroke Patients in Two Groups

A total of forty-six patients were included in the present study. There was no statistically significant difference in the average age, gender ratio, BMI index, hypertension, diabetes mellitus, cardiac disease, and hyperlipidemia between the control group and the chrysanthemum group (*P* > 0.05). NIHSS score was performed on the day of admission in the two groups, and there was no statistically significant difference in NIHSS scores between the two groups (*P* > 0.05), as given in Table 1.

### 3.2. NIHSS Scores and Serum S100 Levels

Severity of stroke in two groups was evaluated by NIHSS score and S100 level on the first and fourth day after treatment. The two-way ANOVA test was used to compare the two groups in terms of NIHSS score (*F* = 8.210, Sig = 0.005) and S100 level (*F* = 10.770, Sig = 0.001) which showed the significant interaction effect between group and time. On the first day after treatment, there was no significant difference in NIHSS score and S100 level between the two groups (*P* > 0.05), as shown in Figure 2. Compared with the first day of treatment, NIHSS score and S100 level in the chrysanthemum group decreased significantly after fourth day of treatment (*P* < 0.05). After fourth day of treatment, NIHSS score and S100 level in the chrysanthemum group were significantly lower than those in the control group (*P* < 0.05). The results show that chrysanthemum extract can effectively reduce the severity of stroke in patients with ischemic stroke.

### 3.3. Serum NSE and BDNF Levels

In order to explore whether chrysanthemum extract has a neuroprotective effect with ischemic stroke patients, we measured the levels of serum neuron related indexes NSE and BDNF on the first and fourth day after treatment. The two-way ANOVA test was used to compare the two groups in terms of NSE (*F* = 10.090, Sig = 0.002) and BDNF levels (*F* = 5.020, Sig = 0.028) which showed the significant interaction effect between group and time. The results showed that after fourth day of treatment, the level of NSE decreased significantly and the level of BDNF increased significantly in both two groups (*P* < 0.05). On the first day after treatment, there was no significant difference in the levels of NSE and BDNF between the two groups (*P* > 0.05). On the 4th day after treatment, the level of NSE decreased significantly and the level of BDNF increased significantly in the chrysanthemum group (*P* < 0.05), as shown in Figure 3. The result suggests that chrysanthemum extract has a neuroprotective effect with ischemic stroke patients.

### 3.4. Serum MDA, SOD, and TAC Levels

The two-way ANOVA test was used to compare the control group and chrysanthemum group in terms of MDA (*F* = 29.210, Sig = 0.000), SOD (*F* = 40.270, Sig = 0.000), and TAC (*F* = 45.730, Sig = 0.000) levels that showed the significant interaction effect between group and time. After one day of treatment, there was no significant difference in the levels of MDA, SOD, and TAC between the chrysanthemum group and the control group (*P* > 0.05). After fourth day of treatment, the level of MDA increased significantly and the levels of SOD and TAC decreased significantly in the control group, and the level of MDA decreased significantly and the levels of SOD and TAC increased significantly in the chrysanthemum group (*P* < 0.05). Compared with the control group, the level of MDA in the chrysanthemum group decreased significantly on the fourth day after treatment, and the levels of SOD and TAC increased significantly (*P* < 0.05), as shown in Figure 4. These results suggest that chrysanthemum extract can effectively improve oxidative stress injury.

## 4. Discussion

Ischemic stroke is caused by cerebral artery stenosis, thrombosis in cerebral artery, or thrombus shedding from other parts blocking cerebral artery [22]. The blood perfusion of local blood supply artery of brain tissue decreases or the blood flow is completely interrupted, and the blood supply, oxygen supply, and sugar supply are stopped, resulting in the disintegration and destruction of local brain tissue [23]. In a short time after ischemic stroke, a large number of neurons still survive in the ischemic penumbra around necrotic brain tissue. The key to save the damaged neurons is to restore the blood perfusion in the ischemic penumbra [24]. However, the reperfusion of blood flow often aggravates the ischemic cascade and causes more serious reperfusion injury of brain tissue, which is the main reason for the high mortality and disability rate of ischemic stroke [25, 26]. There are many pathogenic factors of ischemic stroke. The common causes are vascular diseases, blood system diseases, metabolic diseases, hypertension, coronary heart disease, diabetes, hyperlipidemia, smoking history, and alcoholism [27, 28].

After ischemic occurs, infarction core will release various inflammatory mediators, such as proteases and ROS, which aggravate endothelial damage and necrosis of the tissue [29]. It makes the brain cannot function properly. Cerebral ischemia and reperfusion induce a battery of biochemical and cellular reactions with the generation of excessive ROS. Oxidative stress due to ROS overproduction plays an essential role in the fundamental pathologic progression of brain damage in ischemic stroke [30]. Oxidative stress will occur when the inherent antioxidant potential to neutralize ROS is inadequate and fails to keep the endogenous redox balance. When oxidative stress takes place, ROS can lead to cytotoxicity through oxidative damage of lipids, proteins, and nucleic acids with harmful consequences for the structure and function of cerebral tissue [31, 32]. In ischemic stroke, oxidative stress can also cause neuronal apoptosis, activation of inflammatory signaling pathways, and impairment of the blood-brain barrier (BBB), all of which promote neurodegeneration and cell death [33]. Antioxidant systems include enzymatic antioxidants and nonenzymatic or chemical antioxidants. Enzyme antioxidant substances are generally proteins, such as SOD, which play an important role in the dynamic process of ROS degradation [34]. If too much ROS in cells is not degraded by these substances in time, ROS will accumulate in cells and cause oxidative stress damage.

Neuroprotective agents mainly protect the ischemic penumbra, that is, the survival area around the infarct core, and finally improve the prognosis of patients [35]. Therefore, they are of great significance in the treatment of ischemic stroke. Statins are the most commonly used neuroprotective agents for ischemic stroke [36]. Although there are more and more research and development of neuroprotective drugs, the effectiveness needs to be further confirmed. As one of “the eight genuine traditional Chinese Medicines of Zhejiang” [37], *Chrysanthemum morifolium* may be eaten as food and used as a medicine. *Chrysanthemum morifolium* was recently included in the Chinese Pharmacopoeia (2010 version) [38] and contains flavonoids and triterpenoids as the main active ingredients [39]. In the present study, chrysanthemum extract was used to treat stroke patients, and the changes of clinical indexes, neuronal injury, and oxidative stress indexes were detected after treatment. At present, the indexes to evaluate the severity of stroke patients mainly include the NIHSS score and levels of NSE, S100, and BDNF in serum. NIHSS [40] is widely used to assess the severity of patients with ischemic stroke. Currently, NIHSS is widely used routinely to assess the severity of strokes in stroke service centers. The NIHSS assessment includes eleven components which include level of consciousness, best gaze, visual field testing, facial paresis, arm and leg motor functions, limb ataxia, sensory, language, dysarthria, extinction, and inattention. NIHSS has a maximum score of 42 and a minimum score of 0. The interpretations of NIHSS are score >25 is very heavy, 14–25 severe, 5–14 moderate, and <5 mild. S100 is distributed in a variety of brain cells including blood-brain barrier. It is a specific index of brain tissue injury, can reflect the degree of brain injury, and is a good diagnostic index of stroke [41]. S100 protein specifically exists in glial cells and Schwann cells of the central nervous system, and about 96% of them exist in the brain [42]. In the healthy population, the level of S100 was very low, but after brain injury, the level of S100 in serum and cerebrospinal fluid increased significantly [43]. NSE is mainly distributed in neurons and neuroendocrine cells with high specificity. When neurons are damaged, NSE can leak out of cells into cerebrospinal fluid and blood circulation, increasing the content of NSE in cerebrospinal fluid and blood circulation [44]. The concentration level of NSE in cerebrospinal fluid and serum can reflect the injury and degree of the nervous system, and the increase of NSE level is directly proportional to the degree of neuronal injury [45]. BDNF is a member of neurotrophic factor family. It plays an important role in regulating the development and maturation of the nervous system and maintaining the function of neuronal cells [46]. At the same time, it also has the functions of regulating synaptic plasticity and neurotransmitter transmission. When neurons are damaged and diseased, it is one of the necessary factors to protect their survival and promote their regeneration, so it is also the regulatory factor of neuronal function [47].

Numerous results of the proposed study showed that the use of chrysanthemum extract in the treatment of ischemic stroke patients could significantly reduce the NIHSS score and the levels of S100, NSE, and BDNF in serum, significantly improve the severity of stroke, and reduce the degree of nerve injury. After treatment, the levels of MDA, SOD, and TAC were detected at the same time, suggesting that chrysanthemum extract may improve the severity and nerve injury of stroke patients by improving the degree of oxidative stress. Although the chrysanthemum extract is expected to be effective in such disorders, further more extensive studies are required in this regard.

## 5. Conclusion and Future Work

In this study, we have evaluated the protective effect of chrysanthemum extract on patients with ischemic stroke by detecting the severity of stroke, neuronal indexes, and oxidative stress biomarkers. For this purpose, forty-six patients with ischemic stroke were randomly divided into the control group (*n* = 30) and chrysanthemum group (*n* = 30). The control group received standard stroke treatment, and the chrysanthemum group was treated with chrysanthemum extract 400 mg/day (200 mg/day, twice/day) on the basis of standard treatment. The groups compared the effect of saffron capsules using the National Institute of Health Stoke Scale (NIHSS), serum neuron specific enolase (NSE), S100, brain-derived neurotrophic factor (BDNF), malondialdehyde (MDA), Su-peroxide dismutase (SOD), and total antioxidant capacity (TAC) levels, at the time of first day and fourth day after treatment. On the first day after treatment, there was no significant difference in NIHSS score, serum NSE, S100, BDNF, MDA, SOD, and TAC levels between the chrysanthemum group and the control group (*P* > 0.05). On the fourth day after treatment, the NIHSS, serum NSE, S100, and MDA levels were significantly reduced in the chrysanthemum group compared to the control group, while the BDNF, SOD, and TAC levels were higher (*P* < 0.05). In addition, compared to the levels on the first day, the NIHSS, serum NSE, S100, and MDA levels were significantly reduced, and the BDNF, SOD, and TAC levels were increased in the chrysanthemum group on the fourth day (*P* < 0.05). Chrysanthemum extract has the effects of scavenging oxygen-free radicals and antioxidation and has the neuroprotective effect on ischemic stroke patients.

In future, we are interested to extend the capabilities of the proposed methodology by integrating it with other field proven approaches to form a hybrid scheme which is applicable in different application scenarios.

## Figures and Tables

**Figure 1:** Graphical representation of the proposed model and experimental setup.

**Figure 2:** Severity of stroke evaluated by NIHSS score (a) and S100 (b) level on the first day and fourth day after treatment in the control group and the chrysanthemum group. ^*∗*^*P* < 0.05, compared with the first day of treatment. ^#^*P* < 0.05, compared with the fourth day of treatment in the control group.

**Figure 3:** Levels of neuron related indexes NSE (a) and BDNF (b) in serum detected on the first day and fourth day after treatment in the control group and chrysanthemum group. ^*∗*^*P* < 0.05, compared with the first day of treatment. ^#^*P* < 0.05, compared with the fourth day of treatment in the control group.

**Figure 4:** Levels of serum oxidative stress indexes MDA, SOD, and TAC measured on the first and fourth day after treatment in the control group and chrysanthemum group. ^*∗*^*P* < 0.05, compared with the first day of treatment. ^#^*P* < 0.05, compared with the fourth day of treatment in the control group.

**Table 1:** Clinical characteristics of two groups and their comparisons.

Characteristics	Control group	Chrysanthemum group	*P* value
Age (mean ± SD)	56.13 ± 9.17	58.97 ± 10.06	0.323
Gender (*n*, %)			
Male	15 (65.22)	17 (73.91)	0.522
Female	8 (34.78)	6 (26.09)	
BMI (mean ± SD)	27.49 ± 3.76	28.11 ± 3.95	0.588
Hypertension (*n*, %)	16	17	0.743
Diabetes mellitus (*n*, %)	12	14	0.552
Cardiac disease (*n*, %)	6	5	0.730
Hyperlipidemia (*n*, %)	19	18	0.710
NIHSS (mean ± SD)	9.97 ± 2.49	9.06 ± 2.86	0.256

## Data Availability

The datasets used and analyzed during the current study are available from the corresponding author upon request.
